# Predictive Modeling of Short-Term Poor Prognosis of Successful Reperfusion after Endovascular Treatment in Patients with Anterior Circulation Acute Ischemic Stroke

**DOI:** 10.1155/2022/3185211

**Published:** 2022-08-12

**Authors:** Zhuo Zhang, Cheng Song, Li Zhang, Weimin Yang

**Affiliations:** ^1^Neurointerventional Department, Zhengzhou Central Hospital Affiliated to Zhengzhou University, Zhengzhou 450001, Henan, China; ^2^National Heart and Lung Institute, Imperial College London, London W12 0BZ, UK; ^3^Department of Neurology, The First Affiliate Hospital of Zhengzhou University, Zhengzhou 450052, Henan, China

## Abstract

This study aimed to propose and internally validate a prediction model of short-term poor prognosis in patients with acute ischemic stroke (AIS). In the retrospective study, 356 eligible AIS patients receiving endovascular treatment (EVT) were included and divided into the good prognosis group and the poor prognosis group. Data from 70% of patients were collected as training set and the 30% as validation set. Univariate analysis and multivariate logistic regression were used for identifying independent predictors. The performance of the model was evaluated by receiver operating characteristic (ROC) curve and the paired Chi-square test was used for internal validation. A model for the prediction of short-term poor prognosis in atherosclerotic AIS patients who successfully underwent endovascular reperfusion was developed: log (Pr/1 − Pr) = 3.500 + Blood glucose *∗* 0.174 + Infarct volume *∗* 0.128 + the National Institutes of Health Stroke Scale score × Onset-to-reperfusion time (NIHSS-ORT) *∗* 0.014 + Intraoperative hypotension (Yes) *∗* 1.037 + Mean arterial pressure (MAP) decrease from baseline (>40%) *∗* 2.061 (Pr represented the probability of short-term poor prognosis). The area under the curve (AUC) was 0.806 (0.748 − 0.864) in the training set and 0.850 (0.779 − 0.920) in the testing set, which suggested the good performance of the model. We proposed and validated a combined prediction model to predict the short-term poor prognosis of AIS patients after EVT, which could provide reference for clinicians to identify AIS patients with a higher risk of poor outcomes and thus improving the prognosis of EVT.

## 1. Introduction

Acute ischemic stroke (AIS), the most common type of stroke, has about 72.9% of stroke cases in China [1]. AIS is usually caused by atherosclerotic stenosis, thrombosis, or embolic obstruction, and is characterized by high morbidity, mortality, and recurrence, which requires early intervention [2, 3]. Recently, endovascular treatment (EVT) was a standard and effective treatment for patients with atherosclerotic AIS with significant clinical benefits [4, 5]. However, successful endovascular reperfusion does not guarantee a good prognosis in AIS patients, and the overall probability of comorbidities and ineffectiveness after EVT remains relatively high [6–8]. In view of this, identifying predictors of poor prognosis for AIS patients undergoing EVT are of great significance for timely intervention.

Previous studies have reported that some clinical, biochemical, and imaging factors were associated with poor outcomes of AIS patients after EVT, such as age, the levels of glucose on admission, onset-to-reperfusion time (ORT), onset-to-treatment time (OTT), the National Institutes of Health Stroke Scale (NIHSS) score, neutrophil-lymphocyte ratio (NLR), and the Alberta Stroke Program Early CT Score (ASPECTS) [8–11]. In the study by Todo et al., they indicated that a lower ASPECTS-time score was related to a better clinical outcome for successful reperfusion after EVT in AIS patients [9]. A research group of Wada et al. also reported that the levels of glucose on admission might be an independent predictor of the prognosis for patients after AIS [10]. Nevertheless, it is of particular importance to accurately assess the individual risk probability of AIS patients after receiving EVT and timely give appropriate clinical treatment. To the best of our knowledge, most studies only have investigated the prognostic factors related to AIS patients after EVT so far. Few studies have established an accurate and convenient predictive model by combining multiple prognostic factors for the prediction of outcomes of AIS patients after EVT. Hilbert et al. have investigated the deep learning technique of establishing a model by using CT angiography images to predict the prognosis of good reperfusion after EVT. However, the average AUC of the model was only 0.71 and 0.65 [11]. A single-center study that included 169 patients with atherosclerotic AIS pointed out that they developed a predictive model by a nonconditional logistic stepwise regression analysis for the prediction of the outcome of EVT for patients with atherosclerotic AIS [4]. However, this study excluded some patients with mild and moderate stroke (NIHSS score <7 at admission). A research gap still exists in the prediction of the outcome of EVT for patients with atherosclerotic AIS who were in the entire NIHSS severity range.

Herein, the purpose of this study is to develop a model for the prediction of short-term poor prognosis in atherosclerotic AIS patients who successfully underwent endovascular reperfusion and perform an internal validation to assess its feasibility. In addition, we also evaluated the predictive ability of the established model in patients with different severity of stroke. Thereby helping clinicians identify high-risk population in atherosclerotic AIS, and improving the therapeutic effect and clinical outcomes of EVT in atherosclerotic AIS patients.

## 2. Material and Methods

### 2.1. Patient Population

Totally, 356 atherosclerotic AIS patients who received EVT in the First Affiliated Hospital of Zhengzhou University from September 2019 to September 2020 were enrolled. Inclusion criteria were (1) patients aged ≥18 years old; (2) patients diagnosed with atherosclerotic AIS whose etiology was large artery atherosclerosis; (3) patients with successful reperfusion within 24 hours after clinical evaluation modified treatment in cerebral infarction (mTICI) score ≥2b; and (4) patients with complete clinical data. Exclusion criteria were (1) patients with intracranial hemorrhage or arachnoid hemorrhage detected by CT; (2) patients with malignant tumors, hematological diseases, autoimmune diseases, or infectious diseases; (3) patients with severe heart, liver, or kidney dysfunction; (4) patients with preoperative active infection, including those with pulmonary infection, urinary tract infection, or other obvious typical clinical manifestations such as fever, leukocytosis, or elevated C-reactive protein; (5) patients with active bleeding or significant bleeding tendency; (6) patients whose blood glucose <2.7 mmol/L or >22.2 mmol/L; and (7) patients with severe hypertension that cannot be controlled by drugs. The study has been approved by the Ethics Committee of the First Affiliated Hospital of Zhengzhou University with the approval number 2020-KY-371.

### 2.2. Data Collection

On admission, demographic data of all patients were collected on admission, including age, sex, body mass index (BMI), history of smoking, stroke, and antiplatelet therapy, severity of stroke, level of coma, type of etiology, blood pressure, and comorbidities of diabetes mellitus, hypertension, dyslipidemia, atrial fibrillation, or coronary heart disease. Data from laboratory tests and imaging examinations were also obtained. In addition, data during EVT treatment, including intraoperative blood pressure, NIHSS-ORT (calculated as NIHSS × ORT), and ASPECTS-ORT (calculated as ASPECTS × ORT) were collected. The 3-month follow-ups were conducted in all patients after EVT and a modified Rankin Scale (mRS) score was recorded.

The infarct volume was calculated through the Pullicino formula based on the DWI at admission: *T* (mL) = *π*/6 × *L* (maximum long axis) × *S* (short axis) × Slice (slice thickness, cm). The stroke severity was evaluated by the NIHSS and analyzed by an experienced neurologist; the NIHSS score of 1–4 points was considered as mild stroke, 5–14 points as moderate stroke, 15–24 points as moderate to severe stroke, and ≥25 points as severe stroke [12]. The Glasgow Coma Scale (GCS) is a 3–15-point scale used to describe the level of coma, which is consisted of eye-opening response, verbal response, and motor response; the GCS score of 3–8 points indicates severe coma, 9–12 points indicate moderate coma, and 13–15 points indicate mild coma [13]. The 3-month mRS score was used to evaluate patient prognosis; the mRS score of 0–2 points was considered as good prognosis and the score of 3–6 points as poor prognosis [14].

### 2.3. Treatment Method

Patients underwent EVT after screening for clinical and imaging assessment. The modified Seldinger technology was used to puncture the femoral artery. A 6F arterial sheath and a 5F angiographic catheter were placed for radiography. According to the results, the responsible vessel was confirmed, and whether it was recanalized after EVT and whether the recanalization technique was required were decided. Under general anesthesia, a femoral artery puncture was performed. An 8F arterial sheath and an 8F guide tube were introduced through the occluded segment of the cerebral artery with the help of micro-guide wire and microcatheter. Then we withdrew the wire and introduce a Solitaire stent through the microcatheter. After accurate alignment, the stent was released and slowly recovered 5 minutes later. Then we withdrew the stent and the microcatheter, and removed the thrombus. Repeat angiography was performed to confirm the patency of the cerebral artery, and the modified Thrombolysis in Cerebral Infarction (mTICI) score was calculated. The treatment ended after communication with the family during surgery.

### 2.4. Statistical Analysis

Statistical analyses were performed using SPSS 20.0 software (IBM Co., Armonk, NY, USA) and a two-sided test was adopted for all analyses. Measurement data were analyzed by the Shapiro–Wilk test. For normally distributed variables, the independent samples *t*-test was used for comparison and mean ± standard deviation (mean ± SD) as expression. For non-normally distributed variables, the Mann–Whitney *U* test was carried out for comparison and median and interquartile range (*M* (*Q*1, *Q*3)) as expression. Enumeration data were expressed as case numbers and percentages (*N* (%)), and compared by the Chi-squared test and Fisher's exact test. Data from 70% of patients were selected as the training set and 30% as the validation set. Variables with statistical significance in the univariate analysis were included in the multivariate logistic regression for the development of the prediction model. The receiver operating characteristic (ROC) curve was plotted using Medcalc (Medcalc Software Ltd., Ostend, Belgium) for evaluating the performance of the model. The model was internally validated by the paired Chi-square test, and *P* < 0.05 was considered statistically significant.

## 3. Results

### 3.1. Patient Characteristics

In the present study, 356 patients were enrolled, and divided into the training set (*n* = 248) and the testing set (*n* = 108). In each set, the patients were divided into the poor prognosis group and the good prognosis group. The mean age was 59.37 ± 10.77 years (male: *n* = 230, 64.61%, female: *n* = 126, 35.39%). Based on the NIHSS scores, 133 patients (37.36%) were considered as mild stroke, 209 (58.71%) as moderate stroke, and 14 (3.93%) as stroke with moderate to severe. The GCS results suggested that 25 patients (7.02%) had mild coma and 3 patients (0.84%) had moderate coma. As shown in Table 1, there were no significant differences in all characteristics between the training set and the testing set.

Then, we performed a univariate analysis in the training set. Our results suggested that significant differences were found in NIHSS (*P* < 0.001), the severity of stroke (*P* = 0.001), level of consciousness (*P* < 0.001), basal mean arterial pressure (MAP; *P* < 0.001), basal diastolic blood pressure (DBP; *P* < 0.001), basal systolic blood pressure (SBP; *P* = 0.001), blood glucose (*P* = 0.008), infarct volume (*P* < 0.001), NIHSS-ORT (*P* < 0.001), treatment methods (*P* = 0.041), intraoperative SBP (*P* = 0.031), minimum MAP during operation (*P* < 0.001), intraoperative hypotension (*P* < 0.001), and MAP decreased from baseline >40% between the good and the poor prognosis groups (Table 2).

### 3.2. Independent Predictors of Short-Term Poor Prognosis of AIS Patients After EVT

The above variables that achieved *P* value <0.10 in the univariate analysis were identified and included in the multivariate logistic regression. According to the multivariate analysis, blood glucose, infarct volume, NIHSS-ORT, intraoperative MAP decreased >40% from baseline, and intraoperative hypotension were identified as independent predictors of short-term poor prognosis of AIS after EVT.

For every 1 mmol/L increase in blood glucose, the risk of poor prognosis increased by 0.190-fold (95%CI: 1.037–1.365). The risk of poor prognosis rose by 0.137-fold (95%CI: 1.002–1.290) with every 1 cm^3^ increase in infarct volume. For each unit increase in NIHSS-ORT, the risk increased by 0.014-fold (95%CI: 1.007–1.021). The risk of poor prognosis in patients with intraoperative hypotension was 2.821 times (95%CI: 1.384–5.751) higher than those without. What's more, patients whose intraoperative MAP decreased >40% had a 7.857-fold (95% CI: 2.617–23.587) higher risk of poor prognosis as compared with those ≤40% (Table 3).

### 3.3. Development and Validation of Prediction Model

Then the prediction risk of short-term poor prognosis in atherosclerotic AIS patients was calculated as follow: log (Pr/1 − Pr) = 3.500 + Blood glucose *∗* 0.174 + Infarct volume *∗* 0.128 + NIHSS-ORT *∗* 0.014 + Intraoperative hypotension (Yes) *∗* 1.037 + MAP decrease from baseline (>40%) *∗* 2.061 (Pr represented the probability of short-term poor prognosis). Before determining the final model, we performed the multicollinearity test and the results suggested that no multicollinearity was observed in all predictors (Table 4).

Our ROC curve analyses suggested that the area under the curve (AUC) of the combined model and the single-predictor models (blood glucose, infarct volume, and NIHSS-ORT) were calculated to be 0.806 (95%CI: 0.748–0.864), 0.598 (95%CI: 0.526–0.671), 0.651 (95%CI: 0.583–0.720), and 0.647 (95%CI: 0.576–0.718), respectively. The sensitivities were 0.755 (95%CI: 0.637–0.837), 0.472 (95%CI: 0.377–0.567), 0.849 (95%CI: 0.781–0.917), and 0.613 (95%CI: 0.520–0.706), respectively; the specificities were 0.796 (95%CI: 0.729–0.862), 0.704 (95%CI: 0.629–0.779), 0.380 (95%CI: 0.300–0.460), and 0.690 (95%CI: 0.614–0.766), respectively. The Delong test indicated that the predictive ability of single-factor prediction models, including blood glucose (*Z* = 4.367, *P* < 0.001), infarct volume (*Z* = 3.362, *P* < 0.001), and NIHSS-ORT score (*Z* = 3.393, *P* < 0.001) were all significantly lower compared with the combined model (Figure 1, Table 5).

After the prediction model was developed, we performed an internal validation using data from the testing set. The results showed an AUC of 0.850 (0.779–0.920) with a sensitivity of 0.708 (0.580–0.837) and a specificity of 0.767 (0.660–0.874), which confirmed the good performance of the model (Table 6).

Additionally, in this study, we also assessed the performance of the model in predicting the short-term poor prognosis in atherosclerotic AIS patients after EVT based on different patients with the severity of stroke.  Table 7 suggested that in the training set, the AUC values of model were 0.697 (95%CI: 0.564–0.818) for patients with mild stroke, 0.799 (95%CI: 0.739–0.860) for patients with moderate stroke, and 0.857 (95%CI: 0.548–1.000) for patients with moderate to severe stroke. Similarly, in the testing set, the AUC values of model were 0.905 (95%CI: 0.772–1.000) for patients with mild stroke and 0.836 (95%CI: 0.761–0.911) for patients with moderate stroke.

## 4. Discussion

At present, the efficacy of EVT has been proved in the treatment of AIS patients with large vessel occlusion in the anterior circulation. However, the prognosis of EVT remains to be a problem for the fact that several factors may lead to unfavorable outcomes after successful reperfusion. Most previous studies have used only one or two factors to predict the prognostic outcome of EVT, which may affect the accuracy of prediction. In this study, blood glucose, infarct volume, NIHSS-ORT score, intraoperative MAP decreased >40% from baseline, and intraoperative hypotension were identified as independent predictors using the univariate analysis and multivariate logistic regression analyses. Based on these results, a combined prediction model was developed and internally validated. The prediction risk of short-term poor prognosis in atherosclerotic AIS patients was calculated as follow: log (Pr/1 − Pr) = 3.500 + Blood glucose *∗* 0.174 + Infarct volume *∗* 0.128 + NIHSS-ORT *∗* 0.014 + Intraoperative hypotension (Yes) *∗* 1.037 + MAP decrease from baseline (>40%) *∗* 2.061 (Pr represented the probability of short-term poor prognosis). The ROC analysis demonstrated an AUC of 0.806 and 0.850 suggesting good performance, and the results of the internal validation confirmed the feasibility of the combined model.

To date, previous studies have investigated the independent factors of poor prognosis of AIS after EVT. Our study demonstrated that the blood glucose on admission was independently associated with poor outcomes after EVT. Similarly, Huo et al. reported that higher admission glucose values were associated with poor functional outcomes after EVT [15]. However, another study found there is no association between increased serum glucose on admission and functional outcomes after intra-arterial thrombolysis in patients with AIS due to intracranial proximal arterial occlusion of the anterior circulation [16]. This inconsistency with our results can be explained by the fact that most patients (76%) in Osei's study were normoglycemic, which may affect the accuracy of their conclusions. Moreover, our study did not solely focus on hyperglycemia and included a broader range of admission glucose, which may also lead to this inconsistency. Evidence has shown that a higher level of blood glucose was prone to disrupt the blood-brain barrier, resulting in an increased risk of symptomatic intracerebral hemorrhage, unfavorable functional outcome, and less recanalization after treatment [17–19].

In our study, the NIHSS-ORT score was reported as a predictor of clinical outcomes. Todo et al. [9] demonstrated that the outcomes can be predicted quickly and accurately using the NIHSS-ORT score rather than using the NIHSS score or ORT separately [8]. Studies have also reported that a higher NIHSS score and longer ORT were more likely to be associated with an increased risk of unfavorable outcomes [20, 21], which proves that the NIHSS-ORT score can effectively predict clinical outcomes. In addition, the present study demonstrated infarct volume as an independent predictor. This was consistent with the findings of the previous studies that patients with smaller infarcts showed a lower incidence of reperfusion hemorrhage, and lower mortality [22, 23].

What's more, few studies suggested intraoperative blood pressure as a predictor of the poor prognosis after EVT. However, our results revealed that both intraoperative hypotension and intraoperative MAP decreased >40% from baseline were two predictors of poor prognosis. Similar results were found in another study, which reported that intraoperative hypotension with MAP fall of >40% from baseline was independently associated with poor neurological outcomes [24]. We speculated that anesthetics used for general anesthesia, including propofol or fentanyl for induction, and sevoflurane or remifentanil for maintenance, all had an antihypertensive effect and may lead to intraoperative hypotension. Also, the possible stimulation of the carotid sinus during interventional surgery could cause a significant decrease in blood pressure. In addition, intubation could lead to excessive ventilation and weakening of cerebral autoregulation in patients, which may impair the perfusion of collateral circulation in the ischemic penumbra and therefore affect the prognosis of AIS patients. Therefore, we may suggest that timely monitoring of blood pressure and MAP changes, and being cautious about anesthetic dose and intubation time, may help lower the risk of a significant reduction in blood pressure and MAP during operation, thereby helping to improve the poor prognosis in AIS.

Nowadays, some new technologies were widely used in the risk prediction of diseases, such as a novel knowledge-infused learning framework and an efficient attribute reduction, fuzzy logic classifier [25, 26], and automated machine learning [27]. However, to our knowledge, most previous studies used a single-factor model for predicting the poor outcomes of AIS and few studies were able to set up a combined prediction model. The present study developed a multivariate prediction model, including blood glucose, infarct volume, NIHSS-ORT, intraoperative MAP decreased >40% from baseline, and intraoperative hypotension, and achieved high accuracy. And we also performed an internal validation and the results suggested the feasibility of our model. Moreover, our model also showed a good predictive ability for different patients with the severity of stroke. However, more studies with larger sample sizes will be used to verify the result. In view of this, our multivariate prediction model could effectively predict the short-term prognosis of AIS patients after EVT, which is helpful for clinicians to early identify patients requiring subsequent treatment and follow-up observation, thereby improving the therapeutic effect of EVT as well as the prognosis of AIS patients.

There exist some limitations in the present study. First, this was a single-center retrospective study with small sample size. For lack of data, potential risks of poor prognosis of AIS patients after EVT including symptomatic intracranial hemorrhage, mortality, and long-term risk of restenosis were not discussed here. Second, some other factors such as age were also demonstrated to be associated with the prognosis after EVT, but this association was not significant in our study, which may require multicenter studies with a larger sample size for external validation and for improving the accuracy of our model.

## 5. Conclusions

In the present study, blood glucose, infarct volume, NIHSS-ORT, intraoperative MAP decreased >40% from baseline, and intraoperative hypotension were identified as independent predictors of short-term poor prognosis of AIS patients after EVT. Based on this, we proposed and validated a multivariate prediction model with good performance. It could provide reference for clinicians to identify AIS patients with a higher risk of poor outcomes and thus improving the prognosis of EVT.

## Figures and Tables

**Figure 1:** Receiver operating characteristic curves of prediction models of poor prognosis after EVT.

**Table 1:** Baseline characteristics of all included patients.

Characteristic	Total (*n* = 356)	Dataset		Statistic	*P*
		Training set (*n* = 248)	Testing set (*n* = 108)		
Age, years, Mean ± SD	59.37 ± 10.77	59.86 ± 10.80	58.25 ± 10.69	*t* = 1.30	0.195

Sex, *n* (%)				*χ* ^2^ = 0.087	0.768
Male	230 (64.61)	159 (64.11)	71 (65.74)		
Female	126 (35.39)	89 (35.89)	37 (34.26)		

BMI^*∗*^, kg/m^2^, *n* (%)				*Z* = 0.157	0.875
Underweight	3 (0.84)	3 (1.21)	0 (0.00)		
Normal	158 (44.38)	109 (43.95)	49 (45.37)		
Overweight	168 (47.19)	118 (47.58)	50 (46.30)		
Obese	27 (7.58)	18 (7.26)	9 (8.33)		

Smoking history, *n* (%)				*χ* ^2^ = 1.215	0.270
No	258 (72.47)	184 (74.19)	74 (68.52)		
Yes	98 (27.53)	64 (25.81)	34 (31.48)		

Stroke history, *n* (%)				*χ* ^2^ = 0.035	0.852
No	268 (75.28)	186 (75.00)	82 (75.93)		
Yes	88 (24.72)	62 (25.00)	26 (24.07)		

Antiplatelet therapy history, *n* (%)				*χ* ^2^ = 0.036	0.850
No	258 (72.47)	179 (72.18)	79 (73.15)		
Yes	98 (27.53)	69 (27.82)	29 (26.85)		

Severity of stroke, *n* (%)				*Z* = 1.372	0.170
Mild	133 (37.36)	99 (39.92)	34 (31.48)		
Moderate	209 (58.71)	139 (56.05)	70 (64.81)		
Moderate to severe	14 (3.93)	10 (4.03)	4 (3.70)		

Level of consciousness, *n* (%)				*Z* = 0.183	0.855
No	328 (92.13)	229 (92.34)	99 (91.67)		
Mild	25 (7.02)	16 (6.45)	9 (8.33)		
Moderate	3 (0.84)	3 (1.21)	0 (0.00)		

Baseline blood pressure					
SBP, mmHg, mean ± SD	150.01 ± 24.96	151.21 ± 25.10	147.28 ± 24.55	*t* = 1.37	0.173
DBP, mmHg, mean ± SD	87.44 ± 13.95	87.35 ± 13.53	87.66 ± 14.93	*t* = −0.19	0.847
MAP, mmHg, mean ± SD	108.14 ± 15.69	108.46 ± 15.42	107.41 ± 16.35	*t* = 0.58	0.561

Comorbidities, *n* (%)					
Diabetes mellitus, *n* (%)	120 (33.71)	84 (33.87)	36 (33.33)	*χ* ^2^ = 0.010	0.921
Hypertension, *n* (%)	242 (67.98)	169 (68.15)	73 (67.59)	*χ* ^2^ = 0.011	0.918
Dyslipidemia, *n* (%)	18 (5.06)	13 (5.24)	5 (4.63)	*χ* ^2^ = 0.059	0.808
Coronary heart disease, *n* (%)	56 (15.73)	37 (14.92)	19 (17.59)	*χ* ^2^ = 0.406	0.524

Abbreviations: BMI, body mass index; SBP, systolic blood pressure; DBP, diastolic blood pressure; MAP, mean arterial pressure. ^*∗*^BMI: Underweight (BMI <18.5 kg/m^2^), Normal (18.5 kg/m^2^ ≤ BMI < 24.0 kg/m^2^), Overweight (24 kg/m^2^, BMI < 28.0 kg/m^2^), Obese (BMI ≥ 28 kg/m^2^).18.5 kg/m^2^), Normal (18.5 kg/m^2^ ≤ BMI < 24.0 kg/m^2^), Overweight (24 kg/m^2^ ≤ BMI < 28.0 kg/m^2^), Obese (BMI≥28 kg/m^2^).

**Table 2:** Baseline characteristics of included patients in the training set.

Characteristic	Total (*n* = 248)	Group		Statistic	*P*
		Good prognosis	Poor prognosis		
		(*n* = 142)	(*n* = 106)		
Age, year, (Mean ± SD)	59.86 ± 10.80	58.94 ± 10.90	61.09 ± 10.59	*t* = −1.56	0.121

Sex, *n* (%)				*χ* ^2^ = 0.066	0.797
Male	159 (64.11)	92 (64.79)	67 (63.21)		
Female	89 (35.89)	50 (35.21)	39 (36.79)		

BMI^*∗*^, kg/m^2^, *n* (%)				*Z* = 0.880	0.379
Underweight	3 (1.21)	1 (0.70)	2 (1.89)		
Normal	109 (43.95)	66 (46.48)	43 (40.57)		
Overweight	118 (47.58)	67 (47.18)	51 (48.11)		
Obese	18 (7.26)	8 (5.63)	10 (9.43)		

Smoking history, *n* (%)				*χ* ^2^ = 0.477	0.490
No	184 (74.19)	103 (72.54)	81 (76.42)		
Yes	64 (25.81)	39 (27.46)	25 (23.58)		

Stroke history, *n* (%)				*χ* ^2^ = 0.022	0.882
No	186 (75.00)	106 (74.65)	80 (75.47)		
Yes	62 (25.00)	36 (25.35)	26 (24.53)		

Antiplatelet therapy history, *n* (%)				*χ* ^2^ = 0.020	0.888
No	179 (72.18)	102 (71.83)	77 (72.64)		
Yes	69 (27.82)	40 (28.17)	29 (27.36)		

NIHSS, Mean ± SD	5.00 (4.00, 7.00)	5.00 (3.00, 6.00)	6.00 (4.00, 8.00)	*Z* = 3.981	<0.001

Severity of stroke, *n* (%)				*Z* = 3.179	0.001
Mild	99 (39.92)	68 (47.89)	31 (29.25)		
Moderate	139 (56.05)	71 (50.00)	68 (64.15)		
Moderate to severe	10 (4.03)	3 (2.11)	7 (6.60)		

Level of consciousness, *n* (%)				*Z* = 3.809	<0.001
No	229 (92.34)	139 (97.89)	90 (84.91)		
Mild	16 (6.45)	3 (2.11)	13 (12.26)		
Moderate	3 (1.21)	0 (0.00)	3 (2.83)		

Baseline blood pressure					
SBP, mmHg, Mean ± SD	151.21 ± 25.10	146.82 ± 23.33	157.08 ± 26.26	*t* = −3.24	0.001
DBP, mmHg, Mean ± SD	87.35 ± 13.53	84.70 ± 12.28	90.90 ± 14.34	*t* = −3.66	<0.001
MAP, mmHg, Mean ± SD	108.46 ± 15.42	105.18 ± 13.76	112.85 ± 16.47	*t* = −3.89	<0.001

Comorbidities, *n* (%)					
Diabetes mellitus	84 (33.87)	47 (33.10)	37 (34.91)	*χ* ^2^ = 0.088	0.766
Hypertension	169 (68.15)	94 (66.20)	75 (70.75)	*χ* ^2^ = 0.581	0.446
Dyslipidemia	13 (5.24)	9 (6.34)	4 (3.77)	*χ* ^2^ = 0.804	0.370
Coronary heart disease	37 (14.92)	18 (12.68)	19 (17.92)	*χ* ^2^ = 1.317	0.251

Blood glucose, mmol/L, *M* (*Q*1, *Q*3)	5.36 (4.66, 6.86)	5.21 (4.51, 6.20)	5.77 (4.79, 7.63)	*Z* = 2.651	0.008
HB, g/L, mean ± SD	134.49 ± 17.17	134.46 ± 15.80	134.53 ± 18.93	*t* = −0.03	0.973
RBC, 10^12^/L, mean ± SD	4.36 ± 0.54	4.36 ± 0.53	4.36 ± 0.55	*t* = −0.04	0.964
WBC 10^9^/L mean ± SD	7.07 ± 2.11	6.92 ± 2.07	7.28 ± 2.15	*t* = −1.34	0.181
PLT, 10^9^/L, *M* (*Q*1, *Q*3)	219.50 (177.00, 259.00)	219.00 (176.00, 264.00)	220.50 (179.00, 255.00)	*Z* = −0.064	0.949
NEUT, 10^9^/L, *M* (*Q*1, *Q*3)	4.34 (3.40, 5.40)	4.14 (3.29, 5.19)	4.58 (3.53, 5.61)	*Z* = 1.910	0.056
LYM, 10^9^/L, *M* (*Q*1, *Q*3)	1.66 (1.29, 2.01)	1.69 (1.29, 2.00)	1.56 (1.28, 2.06)	*Z* = −0.889	0.374
NLR, *M* (*Q*1, *Q*3)	2.66 (1.90, 3.56)	2.50 (1.90, 3.28)	2.86 (1.87, 4.34)	*Z* = 1.732	0.083
MONO, 10^9^/L, *M* (*Q*1, *Q*3)	0.46 (0.36, 0.58)	0.45 (0.37, 0.57)	0.46 (0.33, 0.60)	*Z* = 0.053	0.958
TC, mmol/L, *M* (*Q*1, *Q*3)	3.38 (2.75, 4.30)	3.39 (2.67, 4.29)	3.38 (2.80, 4.32)	*Z* = 0.704	0.481
TG, mmol/L, *M* (*Q*1, *Q*3)	1.21 (0.90, 1.68)	1.22 (0.90, 1.75)	1.17 (0.90, 1.65)	*Z* = −0.571	0.568
LDL-C, mmol/L, *M* (*Q*1, *Q*3)	1.92 (1.44, 2.76)	1.85 (1.31, 2.70)	1.96 (1.54, 2.80)	*Z* = 1.089	0.276
HDL-C, mmol/L, Mean ± SD	1.04 ± 0.27	1.05 ± 0.28	1.04 ± 0.24	*t* = 0.25	0.801
CRP, mg/L, *M* (*Q*1, *Q*3)	1.70 (0.93, 3.10)	1.65 (0.92, 2.90)	2.06 (0.98, 5.12)	*Z* = 1.383	0.167
Infarct volume, cm^3^, *M* (*Q*1, *Q*3)	3.10 (2.10, 3.80)	2.75 (1.80, 3.70)	3.55 (2.60, 4.70)	*Z* = 4.074	<0.001
ASPECTS, mean ± SD	7.17 ± 0.88	7.25 ± 0.84	7.08 ± 0.92	*t* = 1.52	0.129
OTT, min, *M* (*Q*1, *Q*3)	320.00 (255.00, 420.00)	320.00 (250.00, 420.00)	315.00 (260.00, 432.00)	*Z* = 0.105	0.917
ORT, min, mean ± SD	771.81 ± 174.17	763.30 ± 165.75	783.21 ± 185.05	*t* = −0.89	0.374
NIHSS-ORT, *M* (*Q*1, *Q*3)	62.84 (44.09, 86.00)	57.33 (42.67, 74.17)	78.00 (48.50, 110.83)	*Z* = 3.956	<0.001
ASPECTS-ORT, mean ± SD	91.83 ± 21.81	91.98 ± 21.95	91.64 ± 21.72	*t* = 0.12	0.901

Treatment methods, *n* (%)				Fisher	0.041
Angioplasty	212 (85.48)	129 (90.85)	83 (78.30)		
Endovascular mechanical thrombectomy	18 (7.26)	7 (4.93)	11 (10.38)		
Thrombus aspiration	14 (5.65)	5 (3.52)	9 (8.49)		
Others	4 (1.61)	1 (0.70)	3 (2.83)		

Intravenous thrombolysis, *n* (%)				*χ* ^2^ = 1.217	0.270
No	234 (94.35)	132 (92.96)	102 (96.23)		
Yes	14 (5.65)	10 (7.04)	4 (3.77)		

Intraoperative blood pressure					
Mean SBP, mmHg, mean ± SD	136.41 ± 20.98	138.88 ± 20.21	133.09 ± 21.61	*t* = 2.16	0.031
Mean DBP, mmHg, mean ± SD	78.63 ± 11.96	79.25 ± 11.51	77.78 ± 12.55	*t* = 0.96	0.339
Intraoperative MAP, mmHg, mean ± SD	97.77 ± 13.53	99.04 ± 12.70	96.06 ± 14.46	*t* = 1.73	0.086
Minimum MAP, mmHg, mean ± SD	82.62 ± 16.21	87.68 ± 14.96	75.85 ± 15.39	*t* = 6.09	<0.001

Intraoperative hypotension, *n* (%)				*χ* ^2^ = 25.305	<0.001
No	167 (67.34)	114 (80.28)	53 (50.00)		
Yes	81 (32.66)	28 (19.72)	53 (50.00)		

MAP decreased from baseline, *n* (%)				*χ* ^2^ = 35.662	<0.001
≤40%	210 (84.68)	137 (96.48)	73 (68.87)		
>40%	38 (15.32)	5 (3.52)	33 (31.13)		

Time when decrease >40%, *M* (*Q*1, *Q*3)	55.00 (29.00, 80.00)	38.00 (30.00, 80.00)	55.00 (29.00, 77.00)	*Z* = 0.000	1.000

Abbreviations: BMI, body mass index; SBP, systolic blood pressure; DBP, diastolic blood pressure; MAP, mean arterial pressure; HB, hemoglobin; RBC, red blood cell; WBC, white blood cell; PLT, platelet; NEUT, neutrophil; LYM, lymphocyte; NLR, neutrophil to lymphocyte ratio; MONO, monocyte; TC, total cholesterol; TG, triglyceride; LDL-C, low-density lipoprotein cholesterol; HDL-C, high-density lipoprotein cholesterol; CRP, C-reactive protein; ASPECTS, Alberta stroke program early CT score; OTT, onset-to-treatment time; ORT, onset-to-reperfusion time; NIHSS, National Institutes of Health Stroke Scale. ^*∗*^BMI: Underweight (BMI <18.5 kg/m^2^), Normal (18.5 kg/m^2^ ≤ BMI < 24.0 kg/m^2^), Overweight (24 kg/m^2^ ≤ BMI <; 28.0 kg/m^2^), Obese (BMI ≥ 28 kg/m^2^).

**Table 3:** Predictors of short-term poor prognosis of AIS after EVT.

Characteristic	*β*	S. E	Wald	*P*	Or (95%CI)
Constant	3.500	0.595	34.632	<0.001	—
Blood glucose	0.174	0.070	6.124	0.013	1.190 (1.037–1.365)
Infarct volume	0.128	0.065	3.948	0.047	1.137 (1.002–1.290)
NIHSS-ORT	0.014	0.004	14.082	<0.001	1.014 (1.007–1.021)

Intraoperative hypotension					
No					Ref
Yes	1.037	0.363	8.146	0.004	2.821 (1.384–5.751)

MAP decrease from baseline					
≤40%					Ref
>40%	2.061	0.561	13.506	<0.001	7.857 (2.617–23.587)

Abbreviations: NIHSS, National Institutes of Health Stroke Scale; ORT, onset-to-reperfusion time; MAP, mean arterial pressure.

**Table 4:** Multicollinearity test for all predictors.

Predictor	Tolerance	VIF
Constant		
Blood glucose	0.999	1.001
Infarct volume	0.956	1.046
NIHSS-ORT	0.947	1.056
Intraoperative hypotension	0.728	1.373
MAP decrease >40% from baseline	0.727	1.375

Abbreviations: VIF, variance inflation factor; NIHSS, National Institutes of Health Stroke Scale; ORT, onset-to-reperfusion time; MAP, mean arterial pressure.

**Table 5:** Predictive efficacy of predictors on short-term prognosis after successful reperfusion in AIS.

Predictor	AUC (95%CI)	SE	Cutoff value	Sensitivity (95%CI)	Specificity (95%CI)	*Z*	*P*
Combine	0.806 (0.748–0.864)	0.030	0.398	0.755 (0.673–0.837)	0.796 (0.729–0.862)		
Blood glucose	0.598 (0.526–0.671)	0.037	0.422	0.472 (0.377–0.567)	0.704 (0.629–0.779)	4.367	<0.001
Infarct volume	0.651 (0.583–0.720)	0.035	0.366	0.849 (0.781–0.917)	0.380 (0.300–0.460)	3.362	<0.001
NIHSS-ORT	0.647 (0.576–0.718)	0.036	0.400	0.613 (0.520–0.706)	0.690 (0.614–0.766)	3.393	<0.001

Abbreviations: AUC, area under the curve; NIHSS, National Institutes of Health Stroke Scale; ORT, onset-to-reperfusion time.

**Table 6:** Predictive efficiency of the validation set.

Parameter	Testing set
AUC (95%CI)	0.850 (0.779–0.920)
Sensitivity (95%CI)	0.708 (0.580–0.837)
Specificity (95%CI)	0.767 (0.660–0.874)
PPV (95%CI)	0.708 (0.580–0.837)
NPV (95%CI)	0.767 (0.660–0.874)

Abbreviations: AUC, area under the curve; PPV, positive predictive value; NPV, negative predictive value.

**Table 7:** Predictive performance of the model based on different patients with the severity of stroke.

Sets	AUC (95%CI)	Sensitivity (95%CI)	Specificity (95%CI)	PPV (95%CI)	NPV (95%CI)
Training set					
Mild stroke	0.691 (0.564–0.818)	0.484 (0.308–0.660)	0.853 (0.769–0.937)	0.600 (0.408–0.792)	0.784 (0.690–0.878)
Moderate stroke	0.799 (0.739–0.860)	0.727 (0.640–0.815)	0.806 (0.740–0.872)	0.727 (0.640–0.815)	0.806 (0.740–0.872)
Moderate to severe stroke	0.857 (0.548–1.000)	1.000 (1.000–1.000)	0.333 (0.000–0.867)	0.778 (0.506–1.000)	1.000 (1.000–1.000)

Testing set					
Mild stroke	0.905 (0.772–1.000)	0.714 (0.380–1.000)	0.963 (0.892–1.000)	0.833 (0.535–1.000)	0.929 (0.833–1.000)
Moderate stroke	0.836 (0.761–0.911)	0.682 (0.544–0.819)	0.767 (0.660–0.874)	0.682 (0.544–0.819)	0.767 (0.660–0.874)
Moderate to severe stroke	1.000 (1.000–1.000)	1.000 (1.000–1.000)	1.000 (1.000–1.000)	1.000 (1.000–1.000)	1.000 (1.000–1.000)

Abbreviations: AUC, area under the curve; PPV, positive predictive value; NPV, negative predictive value.

## Data Availability

The data used to support the findings of this study are available from the corresponding author upon request.
